# The value of serum progesterone level on day of human chorionic gonadotrophin administration / metaphase II oocyte ratio in predicting IVF/ICSI outcome in patients with normal ovarian reserve

**DOI:** 10.1186/s13048-021-00800-5

**Published:** 2021-04-01

**Authors:** Ahmad Mahran, Mohammed Khairy, Reham Elkhateeb, Abdel Rahman Hegazy, Ayman Abdelmeged, Gaber El-Saber Batiha, Khalaf F. Alsharif, Helal F. Hetta, Haitham Ahmed Bahaa

**Affiliations:** 1 Department of Obsterics and Gynecology, Faculty of Medicine, Minia University, Minia, Egypt; 2 Department of Pharmacology and Therapeutics, Faculty of Veterinary Medicine, Damanhour University, Damanhour, Egypt; 3 Department of Clinical laboratory Sciences, College of Applied Medical Sciences, Taif University, Taif, Saudi Arabia; 4 Department of Medical Microbiology and Immunology, Faculty of Medicine, Assiut University, Assiut, Egypt

**Keywords:** Serum progesterone, Metaphase II oocytes, ICSI, Implantation rate, Clinical pregnancy rate

## Abstract

**Background:**

The clinical implication of the increased serum progesterone level on the day of HCG administration in assisted reproduction treatment (ART) is still controversial. The current study aimed to compare the predictive value of serum progesterone on day of HCG administration / metaphase II oocyte (P/MII) ratio on IVF/ ICSI outcome to serum progesterone (P) level alone and the ratio of serum progesterone/estradiol level (P/E2) ratio in prediction of pregnancy rates after ART.

**Material & methods:**

Two hundred patients admitted to the IVF/ICSI program at Minia IVF center in Egypt in the period from October 2016 to May 2018 were included in this study. Serum Progesterone (P) and Estradiol (E2) levels were estimated on the day of HCG administration. The ratio between serum P and the number of MII oocytes (P/MII ratio) was calculated and the predictive values of the three parameters (P, P/E2 ratio and P/MII ratio) in prediction of cycle outcomes were measured.

**Results:**

P/ MII oocyte ratio was significantly lower in patients who attained clinical pregnancy (*n* = 97) as compared with those who couldn’t whilst there was no significant difference in P and P/E2 ratio between the two groups. Using a cut off value of 0.125, the sensitivity and specificity of progesterone/ MII ratio in prediction of no pregnancy in IVF/ICSI were 75.7 and 77.1% respectively with the area under The Receiver operating curve (ROC-AUC) = 0.808. The respective values of the ROC-AUC for the P and P/E2 ratio were 0.651 and 0.712 with sensitivity and specificity of 71.2 and 73.5%for P level and of 72.5 and 75.3% for P/E2 ratio. Implantation or clinical pregnancy rates were significantly different between patients with high and low P/MII ratio irrespective of day of embryo transfer (day 3 or 5).

**Conclusions:**

In patients with normal ovarian response, serum progesterone on day of HCG / MII oocyte ratio can be a useful predictor of pregnancy outcomes and in deciding on freezing of all embryos for later transfer instead of high progesterone level alone.

## Introduction

Current controlled ovarian stimulation (COS) protocols in assisted reproduction treatment (ART) cycles use Gonadotropin-releasing hormone agonists (GnRHa) or antagonists to achieve pituitary down-regulation and to prevent premature luteinizing hormone (LH) surge before oocyte retrieval [1]. Despite that, there is still however a reported subtle elevation of progesterone before triggering ovulation of varied incidence from (5-35) % of stimulated cycles [2–5]. The cause of this premature elevation of progesterone (PE) is still largely unknown. Whilst earlier reports claimed it to be related to premature elevation of LH hence this phenomenon has been known as premature luteinization [6, 7] later reports however have shown it to be related to increased granulosa cells LH receptor and production of Progesterone (P) even in the presence of low LH levels [8–12].

There is a debate about the clinical significance of Premature Progesterone elevation (PE) with a recent systematic review of observational studies showing negative correlation between PE and implantation and clinical pregnancy rates in ART cycles [10]. Proposed mechanism of the detrimental effect of PE on implantation is its impact on endometrial receptivity leading to endometrial glandular/stromal dysregulation and advancement of the implantation window before the embryo transfer [13, 14]. Another postulated mechanism for negative effect of PE is impaired oocyte/embryo quality [15] however reports from oocyte donation and cryopreserved /thawed embryo transfer suggest a more predominant role of PE on endometrial receptivity [16–18]. On the other hand, a negative effect of PE on implantation and pregnancy rates was not shown by many other studies [19–23]. Authors of the latter studies maintain that PE is a reflection of number of recruited follicles and not necessarily a pathological phenomenon.

A common criticism for studies of both views is that they were largely of retrospective nature and failed to adjust for other potential confounders as the age of patients, number of mature oocytes/ high grade embryos, day of embryo transfer, number of embryos transferred as well as to attempt distinguishing between patients with normal and reduced ovarian response to COS.

In fact other studies have attempted to adjust for this shortcoming by studying the progesterone/estradiol ratio (P/E2 ratio) to adjust for number of follicles recruited after COS with reportedly better predictive capacity than absolute P levels [24]. The E2 and P levels however are largely positively correlated and both are thought to exert negative detrimental effect primarily on endometrial receptivity [23].

It has been shown in a large national UK database study that the number of obtained oocytes is one of the most important predictors of clinical pregnancy rate. Relying on progesterone level or P/E2 ratio which are surrogate markers of endometrial receptivity may not be sufficient in predicting the result of IVF/ICSI cycles. Adjusting the ovarian response using the number of available mature oocytes (as a surrogate marker for available embryos) and PE can be more reliable to reflect endometrial receptivity. One study has shown that the Progesterone to follicle index predicted the pregnancy rates more accurately than Progesterone level on the day of HCG trigger did [25]. We have therefore postulated that the Progesterone level/ number of mature metaphase II oocytes (P/MII) ratio would be a better predictor for implantation potential and clinical pregnancy rate in a given ART cycle.

In this study, the impact of PE as defined by absolute P level, P/E2 ratio as well as the P/MII ratio on the implantation and clinical pregnancy rates was prospectively investigated in young patients with normal ovarian reserve.

## Patients and methods

This observational study that included 200 patients undergoing IVF/ICSI treatment in the period from October 2016 to May 2018 at Minia IVF center in Minia, Egypt.

### Eligibility criteria

The inclusion criteria included patients in whom female age ≤ 35 years, baseline day 3 FSH < 10 IU/L, Serum anti-müllerian hormone (AMH) ≥ 1.5 ng/ml, and patients with no prior poor ovarian response defined as ≤4 oocytes retrieved in previous treatment cycles.

We have excluded patients not fulfilling the above criteria as well as if they have any of the following:

- Uterine anomalies or distorted uterine cavity and/or any uterine pathology that could affect implantation as uterine fibroids or known uterine scarring.
- Patients whose male partners required a surgical sperm retrieval procedure.
- Patients with PCOS.

Patient participation was limited to one cycle therefore all patients were represented only once in the study. Both participants in the study and ART practitioners were blinded to the P and E2 levels and this has not influenced decisions regarding freezing embryos, number of embryos transferred, or day of embryo transfer.

Before starting the recruitment, the study was ethically approved by the institutional review board of the faculty of Medicine, Minia University and all the patients were adequately counseled and gave written informed consents.

### Controlled ovarian stimulation protocol

The standard long GnRH agonist protocol for pituitary down regulation was used in all cases. Briefly GnRH agonist in the form of (Decapeptyl, Ferring, USA) was administered at a dose of 0.5 mg by subcutaneous injection from day 21 of the natural cycle preceding the ICSI treatment cycle. Patient had transvaginal ultrasound scan and hormonal assay for E2 on cycle day 1-2 to confirm pituitary down regulation. After pituitary down regulation was confirmed the ovarian stimulation was started with gonadotropins in the form of HMG (Fostimone& Merional, IBSA, Switzerland). The gonadotropin dose was individually modified following to ovarian reserve tests (AMH and antral follicle count (AFC)) and previous response to ovarian stimulation. The GnRH agonist was continued till the day of administration of HCG. Ovarian response was observed with transvaginal ultrasound. Ultrasound scanning began from stimulation day 6 then every other day. Step up or step down protocols were determined according to individual patients’ responses. HCG injection (Choriomone, IBSA, Switzerland) was administrated at a dose of 10.000 IU intramuscular injection when at least 3 follicles larger than 17 mm in diameter were revealed on transvaginal ultrasound scan with the leading follicle approached 18-20 mm in diameter. On the day of HCG administration and before the actual administration patients attended for measurement of their P and E2 levels. Oocytes were obtained under general anesthesia 36 h after HCG administration. Standard procedures as described elsewhere were used [26–29] for ICSI of retrieved oocytes with partner’s sperm, assessment of fertilization and embryos culture. In our center ICSI procedure is used for patients with male factor subfertility, prolonged unexplained, or anovulatory infertility more than 3 years despite normal sperm parameters to minimize incidence of total fertilization failure or low fertilization rates. This led to utilization of ICSI in more than 65% of patients in our center. Embryos were transferred on day 3 after oocyte retrieval for patients with ≤3 grade A embryos on day 3.Patients with > 3 grade A embryos were offered extended culture and transfer on day 5.Grading of embryos on day 3 was done by the morphological assessment criteria described by Van Royen at., 1999 [24] and the criteria described by Schoolcraft and Gardner were used for grading blastocysts on day 5 [29].

All patients had luteal phase support using vaginal 400 mg micronized progesterone (Prontogest, IBSA, Switzerland) suppository BD starting from day of oocyte retrieval till day of pregnancy test. All patients were asked to do a serum pregnancy tests after 14 days of oocyte retrieval and if positive were offered a transvaginal ultrasound to confirm viability and location of pregnancy 2-3 weeks later.

#### Definition of outcomes

Clinical pregnancy was determined as cases who achieved pregnancy with identifiable intrauterine gestational sac, a fetal pole, and visible fetal heart pulsations at 7-8 weeks gestation scan.

Implantation rate was determined as the number of intrauterine gestational sacs identified by ultrasound scan over the number of embryos transferred.

### Hormonal assay

Baseline FSH, LH and AMH were measured between day 2-5 of spontaneous menses in the preceding cycle to ICSI cycle. Serum estradiol (E2) was measured on stimulation cycle day 2 to ensure proper pituitary down-regulation before starting ovarian stimulation and again on HCG day. Serum progesterone (P) was measured once on HCG day. Serum FSH, LH, E2 and P were meaured by (Elecsys 2010; Roche, Germany). The anti Mullerian hormone level was assayed by (AMH Gen II ELISA,Beckman Coulter,USA).

After oocyte retrieval, the number of mature oocytes (MII) was counted and serum P level / number of MII oocytes ratio was calculated. For calculation of the P/E2 level ratio, E2 levels on day of HCG were transformed into Nanogram levels to allow for ratio calculation using unified units of measurements.

### Statistical methodology

All Data on patients’ baseline characteristics (age, Body Mass Index (BMI),type and cause of subfertility, duration of subfertility, previous attempts,baseline ovarian reserve tests),ovarian response and embryological assessment and pregnancy outcomes parameters were prospectively collected and entered onto a spreadsheet and was used for statistical analysis.

Statistical analysis was performed using the Statistical Package for Social Science (SPSS Inc. Chicago) version 21 Microsoft Windows. Data were described in terms of mean ± standard error of mean (SEM) for continuous variables and frequencies and percentages for categorical data. Independent student’s t-test was used to compare quantitative variables and Chi square test was used to compare categorical data. Receiver operator characteristic (ROC) curve analysis was applied to determine the overall performance of different parameters studies as well as to allow for comparison of performance of different parameters. Decision on the thresholds of P, P/E2 ratio and P/MII ratios was based on the value with the optimum sensitivity and specificity of each parameter in prediction of clinical pregnancy as suggested by the ROC curve analysis. A *P* value < 0.05 was considered statistically significant.

## Results

Eligible and consenting patients that were enrolled in the study included 215 patients. A further 15 patients were excluded from the final analysis due to lack of embryo transfer due to either failed fertilization (*n* = 1) or freeze all embryos due to high risk of ovarian hyperstimulation syndrome (*n* = 14). This has led to 200 patients included in the study who had fresh embryo transfer 97 patients (47.5%) achieved clinical pregnancy (Table 1). The number of Patients with elevated progesterone level on the day of HCG administration as defined Progesterone level >  1 ng/ml were (*n* = 120) representing 60% of the cohort studied whilst number of elevated P/E2 ratio > 0.31 were 105 representing 52.5% of the cohort and number of patients with elevated P/MII ratio > 0.125 were 111 representing 55.5% of the cohort.

**Table 1:** Demographic features and baseline hormones in the study population

	Pregnant (***n*** = 97)	Non-pregnant (***n*** = 103)	***P*** value
Age	29.1 ± 0.2	28.8 ± 0.3	0.9
BMI	27.8 ± 0.4	28.1 ± 0.3	0.8
Infertility type:			
-Primary	71 (73.2%)	75 (72.8%)	0.6
-Secondary	26 (26.8%)	28 (27.2%)	0,7
Infertility duration	5.2 ± 0.1	5.4 ± 0.2	0.7
Cause of infertility:			
-Male factor	41	49	0.4
-Tubal factor	22	23	0.8
-Ovulatory factor	7	9	0.4
-Unexplained	27	22	0.5
Basal FSH	5.7 ± 0.6	5.5 ± 0.7	0.8
Basal LH	4.7 ± 0.5	4.4 ± 0.6	0.5
Basal Estradiol(E2) (pg/ml)	37.5 ± 0.6	36.2 ± 0.4	0.9
AMH (ng/ml)	2.7 ± 0.1	2.8 ± 0.2	0.8
AFC	15.5 ± 0.7	16.2 ± 0.9	0.7

Values are presented as mean ± *SEM.FSH* follicle stimulating hormone, *LH* luteinizing hormone, *AMH* anti-müllerian hormone

The receiver operator characteristic (ROC) curve analysis was used to identify the cut off with the best predictive values. A cut off level for P/MII oocyte ratio of 0.125 was associated with a sensitivity of 75.1% and a specificity of 77.1% in predicting pregnancy in IVF/ICSI cycles with area under the curve (AUC) = 0.808 as shown in Fig. 1.

**Fig. 1:** ROC curve analysis of the best cut-off value for P/MII oocyte ratio in prediction of pregnancy after ICSI

The corresponding ROC curve analysis of the best cut-off values for serum progesterone(P-HCG) was 1 ng/ml with sensitivity of 71.2% and specificity of 73.5% and AUC of 0.651 as shown in Fig. 2.

**Fig. 2:** ROC curve analysis of the best cut-off value for serum progesterone on day of HCG in prediction of pregnancy after ICSI

The ROC curve analysis for P / E2 ratio showed an optimum cut off value of 0.31 with sensitivity of 72.5% and specificity of 75.3% and AUC of 0.712 in prediction of Pregnancy after ICSI as shown in Fig. 3.

**Fig. 3:** ROC curve analysis of the best cut-off value for P / E2 ratio on day of HCG in prediction of pregnancy after ICSI

As shown in Table 1, no significant differences were observed between the pregnant and non-pregnant women as regards the personal/clinical baseline characteristics of their infertility and baseline hormonal profiles.

No significant differences were observed regarding the details of controlled ovarian stimulation between the pregnant and non-pregnant women. Serum progesterone on HCG day (P-HCG) and P /E2 ratio were not significantly higher between the pregnant and non-pregnant women. The only significant difference observed was in the serum progesterone/ mature oocyte ratio (P /MII ratio) that was significantly lower in the pregnant women (0.2 ± 0.02 vs 0.36 ± 0.07, *P* < 0.001) as shown in Table 2.

**Table 2:** Details of stimulation cycles and hormonal ratios on HCG day

	Pregnant (***n*** = 97)	Non-pregnant (***n*** = 103)	***P*** value
Gonadotropin dose	2765 ± 37	2870 ± 28	NS
Duration of gonadotropin stimulation	10.5 ± 0.5	11.1 ± 0.4	NS
End. Thickness (mm) on HCG day	10.2 ± 0.04	9.8 ± 0.03	NS
No. of follicles ≥17 mm on HCG day	13.2 ± 0.2	12.9 ± 0.2	NS
Serum P on HCG day (ng/ml)	0.8 ± 0.03	1.7 ± 0.02	NS
Serum Estradiol on HCG day (pglml)	3754.6 ± 73.3	4146.7 ± 64.9	NS
P / E2 ratio	0.21 ± 0.03	0.33 ± 0.04	NS
No. of retrieved oocytes	16.6 ± 0.09	14.1 ± 0.07	NS
N0. of MII oocytes	10.9 ± 1.1	9.7 ± 1	NS
P / MII oocytes ration	0.2 ± 0.02	0.36 ± 0.07	0.001^*^
No of embryos available for transfer	6.2 ± 0.5	6.1 ± 0.2	NS
No. of surplus embryos cryopreserved	3.1 ± 0.2	2.9 ± 0.8	NS
No. of embryos transferred	3.1 ± 0.04	2.9 ± 0.05	NS
No. of grade A embryos transferred	2.8 ± 0.06	2.8 ± 0.05	NS

Values are presented as mean ± SEM. *P* progesterone, *E2* Estradiol, *MII* metaphase II. *NS* non-significant.^*^ Statistically significant

Using the cut off level of P/MII oocyte ratio of 0.125 as determined by the ROC curve, the implantation and clinical pregnancy rates were significantly higher in patients with ratio ≤ 0.125 (29.2, 74.2% respectively as compared with patients with ratio > 0.125 (11.3, 24.3% respectively) with no significant difference in the fertilization rate between the two groups as shown in Table 3. There was no significant difference in implantation and pregnancy rates between patients with low and high P level (28.8%vs 26.3 and 44.2% vs. 36.7% respectively) as well as between patients with low and high P/E2 level (29.1% vs. 27.6 and 49.5%vs 47.6% respectively).

**Table 3:** The differences in embryological/clinical outcomes in relation to different measures of progesterone elevation

	Serum progesterone		***P*** value	P / E2 ratio		***P*** value	P/ MII oocyte ratio		***P*** value
	≤1	> 1		≤0.31	> 0.31		≤0.125	> 0.125	0.84
Fertilization rate	61.2 ± 0.5	62.7 ± 0.7	0.73	60.3 ± 0.4	64.3 ± 0.5	0.62	67.3 ± 0.5	63.7 ± 0.6	0.92
Total no. of embryos transferred	3.1 ± 0.02	2.9 ± 0.0.3	0.81	3.2 ± 0.04	2.9 ± 00.8	0.74	3.1 ± 0.03	3.1 ± 00.1	0.86
No. of grade A embryos transferred	2.6 ± 0.02	2.7 ± 0.0.3	0.81	2.8 ± 0.04	2.7 ± 00.2	0.74	2.7 ± 0.02	2.8 ± 00.3	0.79
Implantation rate	28.8 ± 0.3	26.3 ± 0.4	0.62	29.1 ± 0.2	27.6 ± 0.4	0.85	29.2 ± 0.3	11.3 ± 0.2	0.001*
Clinical pregnancy rate (CPR)	53/80 (44.2%)	44/120 (36.7%)	0.56	47/95 (49.5%)	50/105 (47.6%).	0.79	66/89 (74.2)	27/111 (24.3)	0.001

Values are presented as mean ± SEM.*Statistically significant

In Table 4 we assessed the impact of day of embryo transfer (day3 and day 5) on implantation and pregnancy rates in patients with high vs. low P /MII ratio. In each group, there was no statistically significant difference between patients with high vs low P/MII ratio with regards baseline characteristics, dose of gonadotropins, duration of ovarian stimulation, fertilization rate, number of embryo transferred, and endometrial thickness. There was however a statistically significant difference in the implantation and clinical pregnancy rates between patients with high and low P/MII ratio in each group. In day 3 embryo transfers the implantation and pregnancy rates were 29.3, 75% vs. 12.3,24.7% (*P* < 0.001) between patients with low and high P /MII ratio respectively. Similarly, in day 5 embryo transfers the implantation and pregnancy rates were 31.2, 70.6% vs. 13.3, 22.2% (*P* < 0.001) between patients with low and high P /MII ratio respectively. Miscarriage rate was significantly lower in patients with low P/MII as compared with those with high P/MII 9.3%, 8,3% vs. 17.4, 25%), however multiple pregnancy rates were not significantly different between the two groups.

**Table 4:** Comparison of baseline characteristics and cycle outcomes in patients with high versus low P/MII ratio having day 3 and day 5 embryo transfers

	Day 3 ET		***P*** value	Day 5 ET		***P*** value
	P/MII ≤ 0.125	P/MII > 0.125		P/MII ≤ 0.125	P/MII > 0.125	
No. of cycles	72	93		17	18	
Age	28.3 ± 0.2	29.5 ± 0.3	NS	28.5 ± 0.4	27.8 ± 0.3	NS
BMI (Kg/m^3^)	28.2 ± 0.3	27.1 ± 0.2	NS	27.6 ± 0.3	28.2 ± 0.3	NS
Basal FSH (IU/L)	5.6 ± 0.8	5.5 ± 0.9	NS	5.4 ± 0.1	5.6 ± 0.2	NS
Basal LH (IU/L)	4.3 ± 0.7	4.7 ± 0.5	NS	4.2 ± 0.2	4.4 ± 0.1	NS
AMH (ng/ml)	2.8 ± 0.2	2.6 ± 0.2	NS	2.6 ± 0.3	2.7 ± 0.2	NS
AFC	16.1 ± 0.2	15.8 ± 0.1	NS	15.9 ± 0.4	16.1 ± 0.3	NS
Total gonadotropin dose (IU)	2798.8 ± 75.6	2785.3 ± 82.4	NS	2675.7 ± 87.3	2768 ± 72.4	NS
Duration of gonadotropin stimulation (days)	10.7 ± 0.6	10.9 ± 0.8	NS	11.1 ± 0.2	10.8 ± 0.3	NS
Serum E2 on HCG day	3782.6 ± 87.4	4357 ± 63.8	NS	4123.3 ± 82.4	4232.4 ± 92.3	NS
Endometrial thickness (mm) on HCG day	10.1 ± 0.03	9.9 ± 0.02	NS	9.8 ± 0.1	9.7 ± 0.1	NS
Total no. of embryos transferred	2.8 ± 0.06	3.1 ± 0.07	NS	2.7 ± 0.05	2.6 ± 0..04	NS
No. of High grade embryo/blacytocyst	2.7 ± 0.02	2.7 ± .03	NS	2.6 ± 0.07	2.6 ± 0.02	NS
Fertilization rate	65.6 ± 0.5	63.4 ± 0.6	NS	73.4 ± 0.6	71.3 ± 0.7	NS
Implantation rate	29.3 ± 0.2	12.3 ± 0.3	< 0.001*	31.2 ± 0.3	13.3 ± 0.4	< 0.001*
Clinical pregnancy rate (CPR)	54/72 (75)	23/93 (24.7)	< 0.001*	12/17 (70.6)	4/18 (22.2)	< 0.001*
Miscarriage rate	5/54 (9.3)	4/23 (17.4%)	0.3*	1/12 (8.3%)	1/4 (25%)	0.1*
Multiple pregnancies	19/54 (35.2)	8/23 (34.8%)	0.9	5/12 41.7)	2/4 (50)	0.6

Values are presented as mean ± SEM. NS = non-significant.* statistically significant

## Discussion

This prospective study of patients with normal ovarian reserve having COS and ART demonstrated that isolated P level on the day of HCG administration is not a good predictor of implantation and clinical pregnancy in ART cycles. In our study the P/MII ratio was a more accurate predictor with area under the ROC curve of 0.808 as compared to P level and P/E2 ratio. The usefulness of the (P/MII ratio) is derived from its ability to capture the two main factors affecting implantation i.e. P level as surrogate marker of hormonal milieu affecting endometrial receptivity and MII oocytes as a proxy variable on availability of high grade embryos. The choice of MII oocytes rather than number of follicles prior to HCG trigger or high grade embryos on day of ET was to help inform practice and plan cryopreservation of embryos in timely manner as this was deemed the best compromise in timing and assessment of quality of available cohort of oocytes. The other parameters of P level, P/E2 levels whilst have been reported previously to be predictive of pregnancy outcomes in fresh ART cycles seems to be not informative at least in patients with normal ovarian response and in the presence of large number of high grade embryos. The findings of our study have been suggested previously by other study with similar patient population using three different protocols for pituitary down regulation [30].

In fact, in a recent large report a high progesterone level was not shown to be predictive of lower pregnancy rates while other factors as patient age, day of embryo transfer, number of embryos transferred and number of top quality embryos were shown to be more important in prediction of clinical pregnancy [22]. Another large study elegantly demonstrated that Progesterone level on the day of HCG was not related to pregnancy levels whilst other factors as number of oocytes were shown to be more predictive of clinical pregnancy rates [23]..

Another interesting explanation of lack of predictive capacity of elevated progesterone level is the findings by Shuffaro et al. who postulated that elevated progesterone may be only detrimental if it represents an increased production of progesterone per follicle (i.e increased luteinization of granulosa cells). An elevated progesterone level may therefore be a significant predictor in patients with low ovarian response whilst in patients with large number of follicles it may simply represent a summative effect of normal individual follicle production [16]. The same group has found that the ratio of P level to number of follicles > 14 mm is a better predictor of pregnancy outcomes than the isolated level of progesterone [16].

Other potential explanations for lack of predictive capacity for PE and E2/P ratio seen in our study are;Younger patient population with large number of high quality oocytes retrieved, The use of HMG as main gonadotropin for ovarian stimulation which may have led to lower risk of high progesterone level as has previously reported by other authors [31, 32] and the use of step down protocol in ovarian stimulation may have further lower the incidence of elevated P and E2 levels and reduce the impact of these on endometrial receptivity.

Using the ROC curve analysis we have found that a threshold value of 0.125 for the P/MII ratio to be the optimum trade- off between sensitivity and specificity for prediction of clinical pregnancy to help clinical decision making regarding fresh embryo transfer or freezing all embryos. This ratio level may have been affected by the patient characteristics in this study and may be skewed to higher levels in cohorts with mix of normal and low responders. This would need to be checked in other studies with more representative patient population. It should be noted however that the clinical utility of P/MII ratio may be less in patients with low ovarian reserve who would have higher ratio mainly because of low number of available oocytes (denominator) and not necessarily high level of progesterone. It would therefore seem that high progesterone level alone as denoted by previous studies may be clinically relevant [33]. On the other hand a beneficial effect of adoption of freeze all policy in patients with low number of available embryos has not been proven by randomized clinical trials. A more relevant clinical scenario is in patients with normal ovarian reserve and large number of available embryos who can potentially benefit from freeze all policy hence we included patients with normal ovarian reserve in this study. In this context it would seem that P/MII ratio has more clinical utility than P level only in deciding on embryo transfer policy2 Clearly the adoption of more stringent (higher) ratio levels in freeze all policy may be associated with more specificity (more accurate prediction of negative pregnancy outcomes) however this would lead to lower sensitivity (more patients with negative outcomes after fresh embryo transfer due to inclusion of more patients with imbalance between optimum endometrial receptivity and embryo quality.

The influence of day of embryo transfer (developmental stage of embryo) on the outcome of ART cycles in case of PE or high P/MII ratio was also examined. In our analysis, there was consistently negative effect of high P/MII on the cycle outcomes regardless of the embryo developmental stage (day 3 or 5) in fresh ART cycles therefore it seems that the adverse impact on endometrial receptivity would not be completely rectified by use of day 5 (blastocyst) transfer policy.

The strengths of the current study are its prospective nature and studying of the role of multiple parameters of PE (P level, P/E2 ratio and P/MII ratio) in prediction of ART cycle outcome and its examination of the impact of high P/MII and other PE parameters at different days of embryo transfer as potential remedy for the effect of premature elevation of progesterone.

The limitations of our study are the inclusion of patients with normal ovarian reserve only with majority of patients treated with HMG only. Furthermore our liberal policy of multiple embryos transferred may limit inference on the significant impact of high P level and high P/E2 ratio and generalizability of our findings to other settings using predominantly recombinant FSH for ovarian stimulation and higher proportion of cycles with elective single embryo transfer.

## Conclusion

Serum P/MII oocyte ratio is a good predictor of implantation and clinical pregnancy in fresh ICSI cycles. The findings of this study should help inform clinical management of patients with high P level on the day of HCG. We suggest, based on the findings of this study, that in this scenario the P/MII ratio would be a more helpful parameter to refine criteria of patients who should have cryopreservation of all embryos (elective freeze all policy) and later transfer of cryopreserved/thawed embryo(s). These findings need to be corroborated in other prospective studies, and ideally in randomized clinical trials using high P/MII ratio as main inclusion criterion with randomization to either fresh or frozen embryo transfer.

## Data Availability

Data is available on request.
